# Prediction Model between Serum Vitamin D and Neurological Deficit in Cerebral Infarction Patients Based on Machine Learning

**DOI:** 10.1155/2022/2914484

**Published:** 2022-06-28

**Authors:** Hailiu Zhang, Guotao Yang, Aiqin Dong

**Affiliations:** Department of Neurology, Cangzhou Central Hospital, Cangzhou 061000, China

## Abstract

**Objective:**

Vitamin D is associated with neurological deficits in patients with cerebral infarction. This study uses machine learning to evaluate the prediction model's efficacy of the correlation between vitamin D and neurological deficit in patients with cerebral infarction.

**Methods:**

A total of 200 patients with cerebral infarction admitted to the Department of Neurology of our hospital from July 2018 to June 2019 were selected. The patients were randomly divided into a training set (*n* = 140) and a test set (*n* = 60) in a 7 : 3 ratio. The prediction model is constructed from the training set's data, and the model's prediction effect was evaluated by test set data. The area under the receiver operator characteristic curve was used to assess the prediction efficiency of models.

**Results:**

In the training set, the area under the curve (AUC) of the logistic regression model and XGBoost algorithm model was 0.727 (95% CI: 0.601~0.854) and 0.818 (95% CI: 0.734~0.934), respectively. While in the test set, the AUC of the logistic regression model and XGBoost algorithm model was 0.761 (95% CI: 0.640~0.882) and 0.786 (95% CI: 0.670~0.902), respectively.

**Conclusion:**

The prediction model of the correlation between vitamin D and neurological deficit in patients with cerebral infarction based on machine learning has a good prediction efficiency.

## 1. Introduction

With the improvement of social and economic living standards and the aging of the population, the incidence of acute cerebral infarction is rising [1, 2]. Cerebral infarction has a high disability rate, high mortality rate, and high recurrence rate, which seriously harms the health of the social population and brings a heavy economic burden and medical burden to the family and society [3, 4]. Therefore, the treatment and prevention of stroke to reduce its incidence, mortality, disability rate, and cost of medical treatment has become a fundamental goal of the medical circle.

Vitamin D is a fat-soluble steroid derivative [5]. Vitamin D is hydroxylated in the body to form steroid hormones that regulate metabolism through genomic and nongenomic pathways [6, 7]. In addition to the traditional role of osteoporosis prevention and calcium metabolism [8], a growing number of studies have linked vitamin D deficiency with cardiovascular disease [9], kidney disease, and infections [10]. Vitamin D metabolism and brain diseases are also hot topics. A large number of studies have suggested that low vitamin D levels increase both the incidence of stroke and the incidence of adverse outcomes in stroke patients [11].

The 25-hydroxyvitamin D_3_ (25(OH)D_3_) is an activated vitamin D and is the best indicator of vitamin D levels in the body [12]. In recent years, it has been reported that serum 25(OH)D_3_ level is associated with neurological recovery of acute cerebral infarction, and patients with normal 25(OH)D_3_ levels have a better prognosis than those with 25(OH)D_3_ deficiency [13, 14]. With the development of biomedicine, the application of machine learning in the medical field is increasing gradually [15–17]. Therefore, this study constructed infarction based on machine learning, providing a method for clinical diagnosis and treatment of neurological deficit in patients with cerebral infarction.

## 2. Methods

### 2.1. Research Object

A total of 200 patients with cerebral infarction admitted to the Department of Neurology of our hospital from July 2018 to June 2019 were selected. Inclusion criteria were as follows: (1) clinical diagnosis of acute cerebral infarction: meeting the diagnostic criteria set by the 4th National Academic Conference on Cerebrovascular Diseases and (2) the onset of all patients was within seven days. Exclusion criteria were as follows: (1) patients with severe heart, liver, and kidney diseases; (2) patients with previous neurological diseases and severe sequelae; and (3) patients who took drugs affecting vitamin D metabolism within one week.

### 2.2. Research Methods

Demographic information, past history, personal and family history, and whether patients had taken vitamin D in the last 1 week were collected. All patients underwent blood pressure measurement, nervous system physical examination, and brain imaging examination after admission. Fasting venous blood was taken on the second day of admission to determine the serum 25(OH)D_3_, triglyceride (TG), total cholesterol (TC), low-density lipoprotein (LDL-C), high-density lipoprotein (HDL-C), and other related laboratory indicators. In addition, all subjects were assessed on the National Institute of Health Stroke Scale (NIHSS) on the day of admission. The scale included consciousness, sensation, visual field, gaze, facial paralysis, upper and lower limb movement, ataxia movement, language, and dysarthria. According to their actual situation and physical examination results, the total score of each item is evaluated one by one, which is the NIHSS score of the research object. All the above were carried out under the supervision of physicians with 5 years of clinical experience. Scoring principle is as follows: (1) only the first reaction of the research object is recorded for each item; (2) record the actual ability of the subjects, rather than doctors' subjective opinion; (3) the patients were examined and recorded at the same time without giving any hints to the subjects; and (4) if some items cannot be evaluated, record the highest score of the item. According to NIHSS scoring criteria, NIHSS<7 scores are categorized as mild injury, NIHSS 7-14 scores are categorized as moderate injury, and NIHSS>14 scores are categorized as severe injury.

### 2.3. Machine Learning Model Construction

A data set of 200 patients was randomly divided into a training set (*n* = 140) and a test set (*n* = 60) in a 7 : 3 ratio. Firstly, the training set data is preprocessed to normalize the data. Then, the prediction model is constructed from the data of the training set, and the model is trained. The prediction effect of the model was evaluated by test set data. Then, the predictive efficiency of the model is evaluated. The specific flow chart is shown in Figure 1. Patients in the training set were divided into mild group (*n* = 99), moderate group (*n* = 31), and severe group (*n* = 10) according to the score of the NIHSS.

### 2.4. Construction of Logistic Regression Model

Logistic regression, also known as logistic regression analysis, is a generalized linear predictive regression model often used in data mining, disease diagnosis, and economic forecasting. Logistic regression is the most popular binary data model, and the general logistic regression model has the following forms:

(1) $$\begin{array}{c} \text{Log}\left(\frac{\pi \left(x\right)}{1-\pi \left(x\right)}\right)=\alpha +\beta x. \end{array}$$

The 1-dimensional logistic model has the following form:

(2) $$\begin{array}{c} \text{P}\left(Y=y\right)=\mu^{y}{\left(1-\mu \right)}^{1-y}=\left(1-\mu \right)\exp\left(y\log\frac{\mu }{1-\mu }\right)=\exp\left\{y\theta -\log\left(1+e^{\theta }\right)\right\},\\ y=0,1,\theta =\log\frac{\mu }{1-\mu }. \end{array}$$

The natural connection function is *θ* = *z*′*β*, *μ* = *e*^*z*′*β*^/1 + *e*^*z*′*β*^.

### 2.5. Construction of XGBoost Model

The base learner of the XGBoost algorithm is mainly the classification and regression trees (CART), which can effectively improve the overfitting problem of the single tree model [18]. The main idea is to select some sample features to generate a base learner and continuously fit the previous residuals to minimize the objective function. XGBoost algorithm can be regarded as an additional model composed of *K* trees [19]. The tree model used in this paper is a regression tree, and the specific formula is as follows:

(3) $$\begin{array}{c} {\hat{y}}_{i}=\overset{K}{\underset{K=1}{\sum }}f_{k}\left(x_{i}\right),f_{k}\in F, \end{array}$$

where ${\hat{y}}_{i}$ is the prediction of sample *x*_*i*_, *i* indicates the serial number of the input sample, *K* is the synthesis of threes, and *F* is the set space of all regression trees.

The modeling process of XGBoost keeps the original model unchanged and takes the error generated by the last prediction as a reference to build the next tree.

Initialization:

(4) $$\begin{array}{c} {{\overset{\wedge }{y}}_{i}}^{\left(0\right)}=0. \end{array}$$

Add the first tree to the model:

(5) $$\begin{array}{c} {{\overset{\wedge }{y}}_{i}}^{\left(1\right)}=f_{1}\left(x_{i}\right)={{\overset{\wedge }{y}}_{i}}^{\left(0\right)}+f_{1}\left(x_{i}\right). \end{array}$$

Add the *n*th first tree to the model:

(6) $$\begin{array}{c} {{\overset{\wedge }{y}}_{i}}^{\left(n\right)}=\overset{n}{\underset{k=1}{\sum }}f_{k}\left(x_{i}\right)={{\overset{\wedge }{y}}_{i}}^{\left(n-1\right)}+f_{n}\left(x_{i}\right), \end{array}$$

where ${{\overset{\wedge }{y}}_{i}}^{\left(n\right)}$ is the predicted value of the *i*th sample at the *n*th time, which retains the model prediction result of *n* − 1 time and adds a new function *f*_*n*_(*x*_*i*_). New functions are added in each round to minimize the loss function. At this point, the loss function is

(7) $$\begin{array}{c} L\left(\theta \right)=\overset{n}{\underset{i=1}{\sum }}\text{l}\left(y_{i},{{\overset{\wedge }{y}}_{i}}^{\left(t-1\right)}+f_{t}\left(x_{i}\right)\right). \end{array}$$

First, the clinical data and laboratory results of patients were predicted by logistic regression. Then, the XGBoost model was tuned by adjusting the weight of leaf nodes and the depth of tree model. The XGBoost parameters were adjusted by the fivefold crossover method to obtain the best prediction model, and finally, the feature selection was carried out. The specific process is shown in Figure 2.

### 2.6. Statistical Analysis

SPSS 20.0 software was used for statistical analysis. The measurement data were tested for Shapiro-Wilk normality. The normal distribution was shown by the mean ± standard deviation table, and the nonnormal distribution was expressed by median (interquartile spacing). The Levene method was used to test homogeneity of variance. Bivariate analysis of measurement data: two independent sample *t*-tests were used when normal variance was uniform, *t*-test when normal variance is not uniform, and Wilcoxon rank-sum test for nonnormal distribution. Significance test levels were all *P* < 0.05 which were statistically different.

## 3. Results

### 3.1. Comparison of Clinical Data and Laboratory Results of Patients in Different Sets

Clinical data and laboratory results of patients in the training and test sets were compared. The results showed that there was no significant difference in gender, age, hypertension, diabetes, smoking history, and other laboratory indicators, such as TC, TG, LDL-C, HDL-C, and 25(OH)D_3_ between the two groups (*P* > 0.05). The specific results are shown in Table 1 and Figure 3.

### 3.2. Comparison of 25(OH)D_3_ Levels under Different Neurological Deficit in Training Set

Patients in the training set were divided into mild injury group (*n* = 99), moderate injury group (*n* = 31), and severe injury group (*n* = 10) according to the score of the NIHSS. The serum 25(OH)D_3_ levels in the three groups decreased gradually from the mild group to the severe group, and the differences were statistically significant (*P* < 0.05) (Figure 4).

### 3.3. Evaluation of the Effectiveness of Prediction Models

The area under the receiver operator characteristic (ROC) curve of the logistic regression model in the training set was 0.727 (95% CI: 0.601~0.854). The area under the curve (AUC) of the XGBoost algorithm model is 0.818 (95% CI: 0.734~0.934). In addition, the area under the curve of the logistic regression model in the test set was 0.761 (95% CI: 0.640~0.882). The AUC of the XGBoost algorithm model is 0.786 (95% CI: 0.670~0.902). The detailed ROC curve was shown in Figure 5.

## 4. Discussion

Cerebral infarction refers to the clinical syndrome of cerebral blood supply disorders caused by various reasons, resulting in local cerebral tissue ischemia, hypoxic necrosis, and corresponding neurological defects [20]. Cerebral infarction is one of the three major diseases threatening human health and survival [21]. Cerebral infarction has a high incidence, prevalence, recurrence rate, disability rate, and mortality rate, which brings a great burden to families and society. The majority of cerebral infarction is on the rise in China, which has seriously harmed people's health [22]. Therefore, the treatment and prevention of stroke to reduce its incidence, mortality, disability rate, and lower cost of medical treatment has become a significant goal of the medical circle.

The 25(OH)D_3_ has an extensive biological effect. Besides classic calcium-phosphorus metabolism regulation, anti-inflammatory, immune regulation, lipid metabolism, and cell differentiation, it also inhibits the renin-angiotensin system and affects blood pressure and insulin secretion. This effect can protect target organs such as the heart, blood vessels, lower blood pressure, and blood sugar and slow the hardening of the arteries [23–25]. Recent studies at home and abroad suggest that a low 25(OH)D_3_ level is an independent risk factor for cardiovascular and cerebrovascular diseases [26]. Patients with low 25(OH)D_3_ levels were found to have a significantly increased risk of acute stroke, of which 25(OH)D_3_ was a manageable risk factor [27]. Kiggundu et al. [28] collected 142 patients with acute stroke from a central hospital in Kampala and detected a level of 25(OH)D_3_ in their serum. The results showed that vitamin D deficiency was correlated with stroke. This is consistent with our study, and we found that serum 25 levels were associated with the level of neurological impairment in patients. The serum 25 levels were lowest in patients with severe neurological impairment.

The mechanism of the correlation between serum 25(OH)D3 level and the condition and prognosis of patients with acute ischemic stroke is still unclear. Based on the previous studies, it can be summarized as follows: (1) serum 25(OH)D_3_ has an anti-inflammatory effect, and 25(OH)D_3_ can inhibit endoplasmic reticulum stress during inflammation and reduce the expression of monocyte chemotactic protein 1. This reduces cholesterol deposition in macrophages and ultimately inhibits the formation of atherosclerotic plaques. At the same time, by binding VDR on immune cells to upregulate anti-inflammatory factors, downregulate the expression of inflammatory factors to play an anti-inflammatory effect [29]. (2) Animal experiments have confirmed that serum 25(OH)D_3_ can improve hypercoagulability and antithrombogenesis by downregulating procoagulant tissue factor and upregulating the expression of thrombomodulin [30]. (3) In addition, animal experiments showed that 25(OH)D_3_ had protective effects on focal cerebral ischemia-reperfusion injury, which may be related to reducing oxygen-free radical injury and promoting microvascular regeneration [31]. (4) Atif et al. [32] found that vitamin D can enhance the neuroprotective effect of P4 and reduce the volume of cerebral infarction in the middle cerebral artery infarction model. Vitamin D also regulates the synthesis of neurotransmitters such as acetylcholine, 5-hydroxytryptamine, and dopamine, affecting neurological function.

This study builds a prediction model based on logistic regression and the XGBoost algorithm, and the results show that the area under the curve of the logistic regression model in the test set was 0.761 (95% CI: 0.640~0.882). The area under the curve of the XGBoost algorithm model is 0.786 (95% CI: 0.670~0.902), which shows that the XGBoost model has better prediction performance than logistic regression and can achieve more accurate individual prediction. However, in the training set, there was no significant difference between the two prediction models. The possible reason is that although the XGBoost algorithm model has a unique advantage in dealing with nonlinear relations with high-dimensional variables, the effectiveness of the prediction model is also affected by the nature of variables, sample size, and other factors.

There are some limitations to this study. This study was a single-center cross-sectional retrospective study with a small sample. Further validation is needed in a multicenter prospective study with a large sample. In addition, the effectiveness of the prediction model is affected by the nature and number of variables, which could not play a role in dealing with nonlinear relations.

## 5. Conclusion

The prediction model of the correlation between vitamin D and neurological deficit in patients with cerebral infarction based on machine learning has good prediction efficiency, which can provide a clinical diagnosis and treatment method.

## Figures and Tables

**Figure 1:** Flow chart of machine learning model construction.

**Figure 2:** Flow chart based on logistic regression and XGBoost prediction model.

**Figure 3:** Comparison of clinical data and laboratory results of patients in training set and test set. There was no statistically significant difference between the two sets (*P* > 0.05).

**Figure 4:** Comparison of 25(OH)D_3_ levels in different groups with neurological deficit. ∗: *P* < 0.05.

**Figure 5:** ROC curves of logistic regression model and XGBoost algorithm model in different sets.

**Table 1:** Comparison of clinical data and laboratory results of patients in training set and test set [*n* (%)].

Indicator	Training set (*n* = 140)	Test set (*n* = 60)	*χ* ^2^	*P*
Male	51 (36.4%)	22 (36.7%)	0.001	0.974
Smoking	58 (41.4%)	24 (40.0%)	0.035	0.851
Hypertension	95 (67.9%)	40 (66.7%)	0.027	0.869
Diabetes	45 (32.1%)	19 (31.7%)	0.004	0.947

## Data Availability

The data used to support the findings of this study are available from the corresponding author upon request.
